The article "Research of the Distribution of Tongue Features of Diabetic Population Based on Unsupervised Learning Technology" was published in 2022. Journal: Evid Based Complement Alternat Med.

# Research of the Distribution of Tongue Features of Diabetic Population Based on Unsupervised Learning Technology

**DOI:** 10.1155/2022/7684714

**Published:** 2022-07-05

**Authors:** Jun Li, Longtao Cui, Liping Tu, Xiaojuan Hu, Sihan Wang, Yulin Shi, Jiayi Liu, Changle Zhou, Yongzhi Li, Jingbin Huang, Jiatuo Xu

**Affiliations:** ^1^School of Basic Medicine, Shanghai University of Traditional Chinese Medicine, Shanghai, China; ^2^Shanghai Collaborative Innovation Center of Health Service in Traditional Chinese Medicine, Shanghai University of Traditional Chinese Medicine, Shanghai, China; ^3^Department of Intelligent Science and Technology, Xiamen University, Xiamen, Fujian, China; ^4^China Astronaut Research and Training Center, Beijing, China

## Abstract

**Background:**

The prevalence of diabetes increases year by year, posing a severe threat to human health. Current treatments are difficult to prevent the progression of diabetes and its complications. It is imperative to carry out individualized treatment of diabetes, but current diagnostic methods are difficult to specify an individualized treatment plan.

**Objective:**

Clarify the distribution law of tongue features of the diabetic population, and provide the diagnostic basis for individualized treatment of traditional Chinese medicine (TCM) in the treatment of diabetes.

**Methods:**

We use the TFDA-1 tongue diagnosis instrument to collect tongue images of people with diabetes and accurately calculate the color features, texture features, and tongue coating ratio features through the Tongue Diagnosis Analysis System (TDAS). Then, we used K-means and Self-organizing Maps (SOM) networks to analyze the distribution of tongue features in diabetic people. Statistical analysis of TDAS features was used to identify differences between clusters.

**Results:**

The silhouette coefficient of the K-means clustering result is 0.194, and the silhouette coefficient of the SOM clustering result is 0.127. SOM Cluster 3 and Cluster 4 are derived from K-means Cluster 1, and the intersections account for (76.7% 97.5%) and (22.3% and 70.4%), respectively. K-means Cluster 2 and SOM Cluster 1 are highly overlapping, and the intersection accounts for the ratios of 66.9% and 95.0%. K-means Cluster 3 and SOM Cluster 2 are highly overlaid, and the intersection ratio is 94.1% and 82.1%. For the clustering results of K-means, TB-a and TC-a of Cluster 3 are the highest (*P* < 0.001), TB-a of Cluster 2 is the lowest (*P* < 0.001), and TB-a of Cluster 1 is between Cluster 2 and Cluster 3 (*P* < 0.001). Cluster 1 has the highest TB-b and TC-b (*P* < 0.001), Cluster 2 has the lowest TB-b and TC-b (*P* < 0.001), and TB-b and TC-b of Cluster 3 are between Cluster 1 and Cluster 2 (*P* < 0.001). Cluster 1 has the highest TB-ASM and TC-ASM (*P* < 0.001), Cluster 3 has the lowest TB-ASM and TC-ASM (*P* < 0.001), and TB-ASM and TC-ASM of Cluster 2 are between the Cluster 1 and Cluster 3 (*P* < 0.001). CON, ENT, and MEAN show the opposite trend. Cluster 2 had the highest Per-all (*P* < 0.001). SOM divides K-means Cluster 1 into two categories. There is almost no difference in texture features between Cluster 3 and Cluster 4 in the SOM clustering results. Cluster 3's TB-L, TC-L, and Per-all are lower than Cluster 4 (*P* < 0.001), Cluster 3's TB-a, TC-a, TB-b, TC-b, and Per-part are higher than Cluster 4 (*P* < 0.001).

**Conclusions:**

The precise tongue image features calculated by TDAS are the basis for characterizing the disease state of diabetic people. Unsupervised learning technology combined with statistical analysis is an important means to discover subtle changes in the tongue features of diabetic people. The machine vision analysis method based on unsupervised machine learning technology realizes the classification of the diabetic population based on fine tongue features. It provides a diagnostic basis for the designated diabetes TCM treatment plan.

## 1. Introduction

The number of diabetic patients worldwide is increasing rapidly, posing a major threat to human health [1]. Limited by diagnostic methods, current treatment guidelines are difficult to provide individualized treatment plans. Therefore, existing treatment methods are still difficult to prevent the progression of diabetes and the occurrence and development of complications. Further refined classification of diabetes is conducive to individualized treatment [2]. Syndrome differentiation and treatment of TCM is the practice of individualized treatment. The patient's disease information is collected through tongue diagnosis, pulse diagnosis, and questioning, and the disease is further classified through analysis to formulate an individualized treatment plan [3, 4]. Among them, tongue diagnosis is convenient and noninvasive and can reflect a lot of physiological and pathological information about the human body, so it is an indispensable diagnostic method of TCM [5].

Tongue diagnosis is a classic diagnosis method of TCM. TCM doctors evaluate the disease state by observing changes in tongue body (TB) and tongue coating (TC). They have a long history and rich practical experience. However, on the one hand, due to the influence of light, temperature, humidity, and viewing angle, subtle changes in the color and texture of the tongue require well-trained and experienced physicians to observe. On the other hand, the written tongue diagnosis information is inevitably subjective through visual observation. In order to further improve the standardization and information level of TCM diagnosis, the tongue diagnosis instrument was invented. The tongue diagnosis instrument is equipped with a high-definition camera and a standard light source, which can capture a flat and clear tongue image. It can effectively extract tongue image features with computer image processing technology. These digital tongue features can more accurately characterize the different states of the disease.

Machine learning has been widely used in the field of tongue diagnosis, but the current research focuses on the field of supervised learning, which requires manual calibration of the tongue image [6–8]. It is not difficult to label data with clear diagnostic criteria. However, applying high-dimensional digital tongue features to the classification of the diabetic population is a new research field, and it is difficult to give clear diagnostic criteria, which makes it difficult to explore its internal laws. Unsupervised learning can discover the inherent laws of unlabeled data [9, 10]. Given this, we introduce unsupervised learning technology to study the changing laws of tongue image in different states of the diabetic population and use various methods to evaluate the reliability of the clustering results (Figure 1). Our research will provide an effective analysis method for the classification of the tongue image of diabetes and provide a basis for developing individualized treatment plans.

## 2. Method

### 2.1. Study Population

The subjects participating in our study came from Shuguang Hospital affiliated to Shanghai University of TCM and several Shanghai community hospitals. The data collection period is from August 6, 2018, to December 31, 2019. According to the diagnostic criteria issued by ADA 2020 [11], it is determined that subjects with diabetes have fasting blood glucose ≥ 7.0 mmol/L, blood glucose two hours after a meal ≥ 11.1 mmol/L, or HbA1c ≥ 6.5%. A total of 598 diabetic subjects were included in the study (Table 1). All subjects signed an informed consent form. The study was approved by the IRB of Shuguang Hospital affiliated with Shanghai University of TCM.

### 2.2. Tongue Image Collection and Analysis

The intelligent diagnosis technology research team independently developed the TFDA-1 tongue diagnosis instrument (Figure 2) at the Shanghai University of TCM. It is equipped with a standard light source and a high-definition camera, which can take images of the subject's tongue in a stable light environment. The Tongue Diagnosis Analysis System (TDAS) is used to extract features from tongue images. TDAS can realize the segmentation of tongue body (TB) and tongue coating (TC) [12] and calculate the color feature, texture feature, and tongue coating ratio feature of TB and TC, respectively. Color features include RGB, Lab, YCrCb, and other color space features. In order to facilitate data analysis and interpretation, we chose the color feature of the Lab color space. *L* is used to indicate brightness, the larger the *L* value, the brighter, and vice versa, the darker; a indicates the range from red to green, a positive value indicates red, a higher value indicates red, a negative value indicates green, and a lower value indicates green; *b* indicates the range from yellow to blue, with positive values representing yellow, higher values being more yellow, negative values representing blue, and lower values being blue. Texture features include angular second moment (ASM), entropy (ENT), contrast (CON), and mean (MEAN). ASM has the opposite meaning of ENT, CON, and MEAN. The larger the ASM, the smaller the ENT, CON, and MEAN, and the finer the texture of the tongue, and vice versa. Per-all is inversely proportional to Per-part. The larger the Per-all, the smaller the Per-part, the larger the tongue coating area, and vice versa.

### 2.3. Cluster Analysis

The data analyzed by the clustering algorithm are uncalibrated data. In order to evaluate the reliability of the clustering results, we chose K-means and Self-Organizing Maps (SOM) Network to confirm each other [13, 14]. t-SNE and K-means are implemented and performed in Scikit-learn version 0.23.2 [15].

#### 2.3.1. K-Means Algorithm

Let *X* be the tongue feature and the dimension be *n*; then *X*={*x*_*i*_ : *i*=1, ⋯, *n*}. Let the clustering result be *C* and be divided into *k* clusters; then *C*={*C*_*j*_ : *j*=1, ⋯, *k*} [16].

First, *k* samples {*μ*_1_, *μ*_2_, ⋯, *μ*_*k*_} are randomly selected from *X* as initial cluster centers. Calculate the distance *d*_*ij*_=‖*x*_*i*_ − *μ*_*j*_‖_2_ from the sample *x*_*i*_ to each cluster center *μ*_*j* _(1 < *j* < *k*). The cluster center closest to the sample is recorded as the category of the sample *λ*_*i*_=argmin_*j*∈{1,2, ⋯,*k*}_*d*_*ij*_, and the sample *x*_*i*_ is placed in the corresponding cluster  *C*_*λ*_*i*__=*C*_*λ*_*i*__ ∪ {*x*_*i*_}.

Then calculate the new cluster center *μ*_*j*_′, *μ*_*j*_′=(1/*C*_*j*_)∑_*x*∈*C*_*j*__*x*. If *μ*_*j*_′ ≠ *μ*_*j* _, then update *μ*_*j* _ to *μ*_*j*_′.

The *K*-means algorithm needs to specify the number of clusters *k* value and determine the real *k* value through the elbow method. As the number of clusters *k* increases, the division of clusters becomes more and more refined. The sum of the squared errors (SSE) will gradually become smaller (Equation (1)). When *k* is less than the true number of clusters, the decrease in SSE increases. When *k* is greater than the number of true clusters, the decrease in SSE tends to be flat. The relationship graph between SSE and *k* presents an elbow shape, and the *k* value corresponding to the elbow is the true number of clusters (Figure 3).

(1) $$\begin{array}{c} \text{SSE}=\sum_{i=1}^{k}{\sum_{p\in C_{i}}\left|p-m_{C_{i}}\right|}^{2}, \end{array}$$

where *C*_*i*_ is the *i* cluster, *p* is the sample in *C*_*i*_,  and  *m*_*C*_*i*__ is the mean value of all samples in *C*_*i*_.

#### 2.3.2. SOM Networks

SOM can classify uncalibrated data without additional help. Compared with K-means, there is no need to set the number of categories in advance, and the initial impact is small. Introduce the competitive learning mechanism, and determine the winning neuron by calculating the similarity. The spatial position of the output neuron in the topographic map corresponds to the specific domain or feature drawn from the input space. Finally, the input high-dimensional signal is converted into a two-dimensional discrete map [17].

Let the dimension of tongue feature be *N* and the number of neurons in the computational layer be *M*. Then the tongue feature is expressed as *X*={*x*_*i*_ : *i*=1, ⋯, *N*} and the network weight can be expressed as *W*_*j*_={*w*_*ji*_ : *j*=1, ⋯, *M*; *i*=1, ⋯, *N*}.

Normalize the input vector and network weight:

(2) $$\begin{array}{c} X^{\prime }=\frac{X}{\left\|X\right\|}, \end{array}$$

(3) $$\begin{array}{c} W_{j}^{\prime }=\frac{W_{j}}{\left\|W_{j}\right\|},\;1\;<j\;<M. \end{array}$$

Input the sample into the network, the sample and the weight vector do a dot product, the output neuron with the largest dot product value wins the competition, and it is recorded as the winning neuron.

(4) $$\begin{array}{c} S_{j}=W_{j}\cdot X. \end{array}$$

Update the neurons in the topological neighborhood of the winning neuron, and renormalize the learned weights.

(5) $$\begin{array}{c} \Delta w_{ji}=\eta \left(t\right)\cdot T_{j,I\left(X\right)}\left(t\right)\cdot \left(x_{i}-w_{ji}\right). \end{array}$$

Update the learning rate *η* and the topological neighborhood so that the distance becomes smaller as time increases. If *η* ≤ *η*_min_  or reach the preset number of iterations, the algorithm ends.

t-SNE converts the distance relationship into a probability distribution, which can efficiently perform dimensionality reduction calculations for high-dimensional nonlinear tongue feature data.  Table 2 shows the key parameters we set for the t-SNE algorithm.

### 2.4. Statistical Analysis

The statistical analysis program is coded in Python version 3.8.8. Multiple independent samples are compared using the Kruskal–Willis H test in SciPy version 1.4.1 [18], and the post hoc analyses are performed using the Conover test in Scikit-posthocs 0.6.7 [19]. Machine learning and silhouette coefficient are implemented in Scikit-learn version 0.23.2. Statistical image drawing is implemented in Seaborn version 0.11.1 [20] and Matplotlib version 3.2.2 [21].

(6) $$\begin{array}{c} S=\frac{b-a}{\max\left(a,b\right)}, \end{array}$$

where *a* is the mean distance between a sample and all other points in the same cluster and *b* is the mean distance between a sample and all other points in the next nearest cluster.

## 3. Results

The silhouette coefficient of the K-means clustering result is 0.194, and the silhouette coefficient of the SOM clustering result is 0.127 (Figures 4 and 5). SOM Cluster 3 and Cluster 4 are derived from K-means Cluster 1, and the intersections account for (76.7%, 97.5%) and (22.3%, 70.4%), respectively. K-means Cluster 2 and SOM Cluster 1 are highly overlapped, and the intersection accounts for the ratios are 66.9% and 95.0%. K-means Cluster 3 and SOM Cluster 2 are highly overlapped, and the intersection ratio is 94.1% and 82.1% (Figure 6).

We performed statistical analysis on the clustering results of K-means. Cluster 2 had the highest TB-L and TC-L (*P* < 0.001). Cluster 1 had the lowest TB-L (*P* < 0.05, *P* < 0.001), and Cluster 1 had the lowest TC-L (*P* < 0.001). TB-L of Cluster 3 is between Cluster 1 and Cluster 2 (*P* < 0.05; *P* < 0.001), TB-L of Cluster 3 was between Cluster 1 and Cluster 2 (*P* < 0.05; *P* < 0.001), and the TC-L of Cluster 3 was between Cluster 1 and Cluster 2 (*P* < 0.001) (Figure 7). Cluster 3 had the highest TB-a and TC-a (*P* < 0.001), Cluster 2 had the lowest TB-a (*P* < 0.001), and TB-a of Cluster 1 was between Cluster 2 and Cluster 3 (*P* < 0.001) (Figure 8). Cluster 1 had the highest TB-b and TC-b (*P* < 0.001), Cluster 2 had the lowest TB-b and TC-b (*P* < 0.001), and TB-b and TC-b of Cluster 3 were between Cluster 1 and Cluster 2 (*P* < 0.001) (Figure 9). Cluster 1 had the highest TB-ASM and TC-ASM (*P* < 0.001), Cluster 3 had the lowest TB-ASM and TC-ASM (*P* < 0.001), and TB-ASM and TC-ASM of Cluster 2 were between Cluster 1 and Cluster 3 (*P* < 0.001) (Figure 10). CON, ENT, and MEAN showed the opposite trend (Figures 11–13). Cluster 2 had the highest Per-all (*P* < 0.001). The Per-part of Cluster 2 was the lowest (*P* < 0.001), the Per-part of Cluster 3 was the highest (*P* < 0.01, *P* < 0.001), and the Per-part of Cluster 1 was between Cluster 2 and Cluster 3 (*P* < 0.01; *P* < 0.001) (Figure 14).  Figure 15 shows the representative tongue images in the three groups.

SOM divides K-means Cluster 1 into two categories. Through statistical analysis, it was found that there was almost no difference in texture features between Cluster 3 and Cluster 4 of SOM. Cluster 3's TB-L, TC-L, and Per-all were lower than Cluster 4 (*P* < 0.001), Cluster 3's TB-a, TC-a, TB-b, TC-b, and Per-part were higher than Cluster 4 (*P* < 0.001) (Figure 16 and Table 3).  Table 4 shows the results of the statistical analysis of the laboratory tests based on K-means clustering.  Table 5 shows the results of the statistical analysis of the laboratory tests based on SOM clustering.

## 4. Discussion

In order to comprehensively and objectively characterize the tongue image, the tongue features extracted by the TDAS include high-dimensional structural data such as color features, texture features, and tongue coating ratio features. These fine tongue features describe tongue changes from multiple angles and explain the tiny differences in tongue features of different states of disease. It is difficult for us to use manual observation and general statistical methods to measure the internal correlation of tongue features and specify diagnostic criteria. Clustering algorithms group samples with similar characteristics into a group through repeated iterations, and are often used to identify outliers, explore the inherent laws of complex data, and make predictions [22, 23].

An adequate evaluation of the clustering results is necessary for reaching a reliable conclusion. We take many measures to evaluate the clustering results. Firstly, K-means and SOM are used to calculate the results of two completely different clustering algorithms and confirm each other. Through the t-SNE algorithm and Venn diagram to visually analyze the clustering results, K-means Clusters and SOM Clusters are highly overlapping. Next, through statistical analysis, it is found that there are extremely significant differences in the tongue features between the clusters, which proves that the differences between the clusters are extremely large. Finally, by displaying the representative tongue samples of each cluster, itis found that the differences are visible to the naked eye.

The classification of the diabetic population based on the tongue features provides a new understanding of the heterogeneity of diabetes. We found that the tongues of people with diabetes are divided into three types through cluster analysis. The first type of tongue is characterized by a red tongue and a dry and rough tongue; the second type of tongue is characterized by a purple tongue and a large and thick tongue coating; the third type of tongue is mainly characterized by its fine texture. Chinese medicine believes that the first tongue is a sign of heat syndrome, the second tongue is a sign of phlegm and blood stasis, and the third tongue is a sign of deficiency syndrome. The above classification is expected to provide an objective basis for the individualized treatment of diabetes and has potential clinical value. K-means divides the diabetic population into 3 categories, while SOM divides the diabetic population into 4 categories, of which two clusters are highly overlapping. SOM subdivides one cluster in K-means into two categories. The difference between the two categories is mainly reflected in the color features and coating ratio features. Our research proves that digital tongue features can characterize subtle changes in the tongue of diabetic people. High-precision image measurement technology combined with unsupervised machine learning technology is the key means to discover this difference.

Our research found that machine vision can keenly perceive the subtle changes in the tongue of diabetic patients and realize the fine classification of the diabetic population, providing a diagnosis basis for the individualized treatment of diabetes in TCM. We verify each other through two clustering algorithms with completely different mechanisms. Statistical analysis, t-SNE, Venn diagram visualization analysis, and tongue image examples fully prove the reliability of the clustering results. However, our data lack information on the course of the disease, and it is impossible to further infer the evolutionary law of tongue features in the course of diabetes.

## 5. Conclusion

The fine tongue features calculated by TDAS are the basis for classifying the diabetic population. We have discovered the inherent law of tongue features of people with diabetes through unsupervised machine learning technology. The application of statistical analysis to compare the differences between the clusters clarified the meaning of the tongue features of each cluster. Our study laid the foundation for implementing individualized treatment of diabetes in TCM. In the future, we will expand the sample size and build a standard tongue feature database for diabetic population classification.

## Figures and Tables

**Figure 1:** Work flow.

**Figure 2:** TFDA-1 tongue diagnosis instrument.

**Figure 3:** Elbow diagram.

**Figure 4:** Visualization of *K*-means clustering results based on t-SNE algorithm.

**Figure 5:** Visualization of SOM clustering results based on t-SNE algorithm.

**Figure 6:** Venn diagram of clustering results of *K*-means and SOM.

**Figure 7:** TB-L and TC-L of *K*-means clustering results.

**Figure 8:** TB-a and TC-a of *K*-means clustering results.

**Figure 9:** TB-b and TC-b of *K*-means clustering results.

**Figure 10:** TB-ASM and TC-ASM of *K*-means clustering results.

**Figure 11:** TB-CON and TC-CON of *K*-means clustering results.

**Figure 12:** TB-ENT and TC-ENT of *K*-means clustering results.

**Figure 13:** TB-mean and TC-mean of *K*-means clustering results.

**Figure 14:** Per-all and per-part of *K*-means clustering results.

**Figure 15:** Examples of tongue images of *K*-means' 3 clusters. Note. To the naked eye, there are significant differences between the three types of tongue images. (a) Cluster 1 has the most delicate texture, (b) Cluster 2 has the most purple color, and (c) Cluster 3 has the roughest texture.

**Figure 16:** Tongue feature distribution based on SOM algorithm.

**Table 1:** Dataset description.

Class	Item	Mean ± SD/median (P_25_, P_75_)
Basic information	Male (%)	357 (59%)
	Age (years)	58.00 (49.00, 63.00)

Glucose and lipid metabolism	GLU (mmol/L)	7.22 (6.05, 8.50)
	HbA1c (%)	6.75 (6.50, 7.40)
	TCHO (mmol/L)	5.20 (4.54, 5.92)
	TG (mmol/L)	1.79 (1.25, 2.61)
	LDL (mmol/L)	2.91 ± 0.96
	HDL (mmol/L)	1.20 (1.03, 1.41)

Liver function	ALT (U/L)	23 (16, 38)
	AST (U/L)	21 (17, 29)
	GGT (U/L)	32 (21, 51)

Kidney function	UA (umol/L)	338 (287, 411)
	CREA (umol/L)	69 (58, 80)
	BUN (mmol/L)	5.19 (4.47, 6.08)

*Note.* Laboratory results included the following: (1) glucose and lipid metabolism including blood glucose (GLU), glycosylated hemoglobin (HbA1c), total cholesterol (TCHO), triglycerides (TG), low-density lipoprotein (LDL), and high-density lipoprotein (HDL); (2) liver function including alanine aminotransferase (ALT), aspartate transaminase (AST), and gamma-glutamyl transpeptidase (GGT); (3) kidney function including uric acid (UA), creatinine (CREA), and blood urea nitrogen (BUN).

**Table 2:** Key parameters of t-SNE.

Parameter	Value
Perplexity	30
Early_exaggeration	12
Learning_rate	200
N_iter	1000
Min_grad_norm	1*e*−7
Metric	Euclidean
Method	Barnes–Hut

**Table 3:** Tongue feature comparation based on SOM 4 clusters.

Item	Cluster 1	Cluster 2	Cluster 3	Cluster 4
TB-L	49.905 (47.923, 51.967)	47.959 (46.683, 49.431) ^*∗*^ ^*∗*^ ^*∗*^	47.057 (45.501, 48.402)^###▲▲▲^	48.706 (47.468, 50.538)^△□□☆☆☆^
TB-a	23.918 (22.537, 25.220)	27.014 (25.663, 28.404) ^*∗*^ ^*∗*^ ^*∗*^	27.660 (25.975, 28.907)^###▲^	23.780 (22.818, 25.239)^□□□☆☆☆^
TB-b	5.949 (4.614, 6.866)	7.999 (7.065, 9.162) ^*∗*^ ^*∗*^ ^*∗*^	9.174 (8.118, 10.371)^###▲▲▲^	7.478 (6.750, 9.075)^△△△☆☆☆^
TC-L	53.518 (50.644, 55.435)	51.717 (49.192, 53.752) ^*∗*^ ^*∗*^ ^*∗*^	46.691 (43.692, 49.318)^###▲▲▲^	51.142 (49.669, 52.920)^△△△☆☆☆^
TC-a	15.905 ± 1.915	18.518 ± 2.043 ^*∗*^ ^*∗*^ ^*∗*^	19.220 ± 2.189^###▲▲^	16.948 ± 1.833^△△△□□□☆☆☆^
TC-b	3.575 ± 2.035	5.304 ± 1.863 ^*∗*^ ^*∗*^ ^*∗*^	6.590 ± 1.854^###▲▲▲^	5.730 ± 1.811^△△△☆☆☆^
TB-CON	80.025 (70.801, 92.922)	91.638 (80.664, 110.948) ^*∗*^ ^*∗*^ ^*∗*^	53.213 (45.052, 63.684)^###▲▲▲^	51.768 (44.479, 58.037)^△△△□□□☆^
TB-ASM	0.072 (0.066, 0.077)	0.068 (0.062, 0.074) ^*∗*^ ^*∗*^	0.091 (0.082, 0.100)^###▲▲▲^	0.092 (0.085, 0.101)^△△△□□□^
TB-ENT	1.238 (1.212, 1.275)	1.268 (1.236, 1.310) ^*∗*^ ^*∗*^ ^*∗*^	1.143 (1.096, 1.188)^###▲▲▲^	1.134 (1.101, 1.164)^△△△□□□^
TB-MEAN	0.027 (0.026, 0.029)	0.029 (0.027, 0.032) ^*∗*^ ^*∗*^ ^*∗*^	0.022 (0.020, 0.024)^###▲▲▲^	0.022 (0.020, 0.023)^△△△□□□^
TC-CON	96.448 (82.107, 107.996)	125.628 (109.574, 149.131) ^*∗*^ ^*∗*^ ^*∗*^	60.078 (48.983, 72.450)^###▲▲▲^	65.916 (55.146, 74.215)^△△△□□□^
TC-ASM	0.064 (0.060, 0.072)	0.055 (0.050, 0.060) ^*∗*^ ^*∗*^ ^*∗*^	0.084 (0.075, 0.094)^###▲▲▲^	0.080 (0.073, 0.087)^△△△□□□^
TC-ENT	1.282 (1.245, 1.306)	1.343 (1.312, 1.381) ^*∗*^ ^*∗*^ ^*∗*^	1.166 (1.125, 1.218)^###▲▲▲^	1.194 (1.152, 1.225)^△△△□□□^
TC-MEAN	0.030 (0.028, 0.032)	0.035 (0.032, 0.037) ^*∗*^ ^*∗*^ ^*∗*^	0.024 (0.021, 0.026)^###▲▲▲^	0.025 (0.023, 0.027)^△△△□□□^
Per-all	0.456 (0.429, 0.481)	0.341 (0.297, 0.400) ^*∗*^ ^*∗*^ ^*∗*^	0.303 (0.250, 0.363)^###▲▲▲^	0.422 (0.400, 0.468)^△□□□☆☆☆^
Per-part	1.076 (1.042, 1.132)	1.188 (1.099, 1.363) ^*∗*^ ^*∗*^ ^*∗*^	1.190 (1.106, 1.338)^###^	1.112 (1.044, 1.177)^□□□☆☆☆^

^*∗*^denotes the comparison of Cluster 1 and Cluster 2,  ^*∗*^*P* < 0.05,  ^*∗*^ ^*∗*^*P* < 0.01, and  ^*∗*^ ^*∗*^ ^*∗*^*P* < 0.001.^#^ denotes the comparison of Cluster 1 and Cluster 3, ^#^*P* < 0.05,^##^*P* < 0.01, and ^###^*P* < 0.001. ^△^ denotes the comparison of Cluster 1 and Cluster 4, ^△^*P* < 0.05, ^△△^*P* < 0.01, and ^△△△^*P* < 0.001. ^▲^ denotes the comparison of Cluster 2 and Cluster 3, ^▲^*P* < 0.05, ^▲▲^*P* < 0.01, and ^▲▲▲^*P* < 0.001. ^□^ denotes the comparison of Cluster 2 and Cluster 4, ^□^*P* < 0.05, ^□□^*P* < 0.01, and ^□□□^*P* < 0.001. ^☆^ denotes the comparison of Cluster 3 and Cluster 4, ^☆^*P* < 0.05, ^☆☆^*P* < 0.01, and ^☆☆☆^*P* < 0.001.

**Table 4:** Laboratory results (*K*-means).

Item	Cluster 1 (*n* = 256)	Cluster 2 (*n* = 172)	Cluster 3 (*n* = 170)
Gender (*n*, %)	144 (56)	112 (65)	86 (51)

Age (years)	57 (49, 63)	57 (49, 63)	60 (52, 65)^☆★^

GLU (mmol/L)	7.300 (6.215, 8.412)	7.480 (6.395, 9.045)	6.845 (5.592, 8.100)^☆★★^
	(*n* = 256)	(*n* = 171)	(*n* = 170)

TCHO (mmol/L)	5.306 ± 1.106	5.284 ± 1.066	5.118 ± 1.051
	(*n* = 244)	(*n* = 163)	(*n* = 164)

TG (mmol/L)	1.730 (1.240, 2.420)	1.920 (1.330, 2.960)	1.660 (1.222, 2.468)
	(*n* = 244)	(*n* = 163)	(*n* = 164)

LDL (mmol/L)	2.935 (2.328, 3.652)	2.915 (2.260, 3.485)	2.890 (2.165, 3.485)
	(*n* = 212)	(*n* = 134)	(*n* = 147)

HDL (mmol/L)	1.185 (1.050, 1.455)	1.190 (1.002, 1.300)	1.230 (1.030, 1.400)
	(*n* = 212)	(*n* = 134)	(*n* = 147)

UA (umol/L)	333.500 (280.750, 412.750)	341.000 (288.000, 421.000)	346.500 (293.750, 399.750)
	(*n* = 256)	(*n* = 171)	(*n* = 170)

ALT (U/L)	23.000 (15.000, 40.000)	24.000 (16.500, 35.500)	24.000 (15.250, 38.000)
	(*n* = 256)	(*n* = 171)	(*n* = 170)

AST (U/L)	21.000 (17.000, 30.000)	21.000 (17.000, 27.000)	21.000 (18.000, 29.000)
	(*n* = 252)	(*n* = 167)	(*n* = 169)

GGT (U/L)	31.000 (21.000, 51.750)	35.500 (24.250, 51.750)	31.000 (21.000, 46.000)
	(*n* = 250)	(*n* = 162)	(*n* = 161)

TBIL (umol/L)	12.400 (9.000, 16.200)	13.000 (10.350, 16.775)	11.400 (9.400, 15.500)
	(*n* = 221)	(*n* = 146)	(*n* = 141)

CREA (umol/L)	68.500 (57.000, 80.000)	71.000 (60.000, 80.000)	70.000 (59.000, 80.000)
	(*n* = 256)	(*n* = 171)	(*n* = 170)

BUN (mmol/L)	5.055 (4.400, 6.000)	5.275 (4.500, 6.250)	5.190 (4.600, 6.000)
	(*n* = 254)	(*n* = 170)	(*n* = 170)

eGFR (ml/min*∗*1.73 m^2)	107.900 (92.200, 121.100)	104.220 (92.240, 117.500)	101.000 (86.000, 114.900)
	(*n* = 217)	(*n* = 137)	(*n* = 138)

^☆^denotes the comparison of Cluster 1 and Cluster 3, ^☆^*P* < 0.05, ^☆☆^*P* < 0.01, and ^☆☆☆^*P* < 0.001. ^★^ denotes the comparison of Cluster 2 and Cluster 3, ^★^*P* < 0.05, ^★★^*P* < 0.01, and ^★★★^*P* < 0.001.

**Table 5:** Laboratory results (SOM).

Item	Cluster 1 (*n* = 121)	Cluster 2 (*n* = 195)	Cluster 3 (*n* = 201)	Cluster 4 (*n* = 81)
Gender (*n*, %)	82 (68)	99 (51)	112 (56)	49 (60)

Age (years)	56 (48, 62)	61 (54, 65) ^*∗*^ ^*∗*^	57 (50, 63)^▲^	54 (46, 61)^□□□^

GLU (mmol/L)	7.565 (6.360, 9.250)	6.900 (5.585, 8.100) ^*∗*^ ^*∗*^	7.200 (6.330, 8.240)	7.810 (6.300, 9.670)^□□^
	(*n* = 120)	(*n* = 195)	(*n* = 201)	(*n* = 81)

TCHO (mmol/L)	5.376 ± 1.128	5.061 ± 1.022	5.296 ± 1.084	5.384 ± 1.098
	(*n* = 114)	(*n* = 189)	(*n* = 192)	(*n* = 76)

TG (mmol/L)	1.935 (1.397, 2.860)	1.610 (1.200, 2.420)	1.745 (1.240, 2.433)	1.975 (1.488, 2.832)
	(*n* = 114)	(*n* = 189)	(*n* = 192)	(*n* = 76)

LDL (mmol/L)	2.960 (2.230, 3.580)	2.790 (2.210, 3.370)	2.940 (2.335, 3.570)	2.990 (2.310, 3.705)
	(*n* = 95)	(*n* = 167)	(*n* = 164)	(*n* = 67)

HDL (mmol/L)	1.190 (1.025, 1.365)	1.230 (1.020, 1.440)	1.180 (1.048, 1.450)	1.110 (1.025, 1.325)
	(*n* = 95)	(*n* = 167)	(*n* = 164)	(*n* = 67)

UA (umol/L)	345.(294, 419)	337 (292, 401)	340 (287, 412)	326 (253, 422)
	(*n* = 120)	(*n* = 195)	(*n* = 201)	(*n* = 81)

ALT (U/L)	25 (17, 38)	23 (16, 36)	23 (16, 40)	24 (15, 35)
	(*n* = 120)	(*n* = 195)	(*n* = 201)	(*n* = 81)

AST (U/L)	21 (18, 29)	21 (18, 28)	21 (17, 30)	20 (17, 29)
	(*n* = 119)	(*n* = 191)	(*n* = 198)	(*n* = 80)

GGT (U/L)	36 (24, 53)	31 (21, 44)	31 (21, 53)	37 (24, 57)
	(*n* = 115)	(*n* = 182)	(*n* = 195)	(*n* = 81)

TBIL (umol/L)	13 (11, 17)	12 (9, 16)	12 (9, 16)	13 (9, 17)
	(*n* = 104)	(*n* = 161)	(*n* = 173)	(*n* = 70)

CREA (umol/L)	72 (61, 80)	70 (59, 81)	68 (56, 79)	71 (57, 80)
	(*n* = 120)	(*n* = 195)	(*n* = 201)	(*n* = 81)

BUN (mmol/L)	5.295 (4.470, 6.455)	5.120 (4.518, 5.975)	5.100 (4.415, 6.000)	5.000 (4.450, 6.100)
	(*n* = 120)	(*n* = 194)	(*n* = 199)	(*n* = 81)

eGFR (ml/min*∗*1.73 m^2)	104 (93, 117)	102 (87, 117)	107 (91, 122)	103 (92, 115)
	(*n* = 99)	(*n* = 155)	(*n* = 170)	(*n* = 68)

*∗* denotes the comparison of Cluster 1 and Cluster 2,  ^*∗*^*P* < 0.05,  ^*∗*^ ^*∗*^*P* < 0.01, and  ^*∗*^ ^*∗*^ ^*∗*^*P* < 0.001. ^▲^ denotes the comparison of Cluster 2 and Cluster 3, ^▲^*P* < 0.05, ^▲▲^*P* < 0.01, and ^▲▲▲^*P* < 0.001. ^□^ denotes the comparison of Cluster 2 and Cluster 4, ^□^*P* < 0.05, ^□□^*P* < 0.01, and ^□□□^*P* < 0.001.

## Data Availability

The experimental data used to support the findings of this study were supplied by Prof. Jiatuo Xu under license and thus cannot be made freely available. Requests for access to these data should be made to Prof. Jiatuo Xu (e-mail: xjt@fudan.edu.cn).
